The article "Clinical Observation of Intraosseous Anesthesia in Percutaneous Kyphoplasty" was published in 2021. Journal: J Healthc Eng.

# Clinical Observation of Intraosseous Anesthesia in Percutaneous Kyphoplasty

**DOI:** 10.1155/2021/5528073

**Published:** 2021-06-01

**Authors:** Li-Shuai Bao, Wei Wu, Xin Wang, Xi-Hong Zhong, Lin-Xiu Wang, Hong Wang

**Affiliations:** ^1^The Second Affiliated Hospital of Chengdu Medical College (China National Nuclear Corporation 416 Hospital), Chengdu 610000, China; ^2^Clinical Medical College & Affiliated Hospital of Chengdu University, Chengdu 610000, China; ^3^The First Affiliated Hospital of Dalian Medical University, Dalian 116000, China; ^4^Dalian Municipal Central Hospital, Dalian, China

## Abstract

**Objective:**

Percutaneous kyphoplasty (PKP) is an effective minimally invasive technique in spine surgery in recent years. General anesthesia and local anesthesia are the main ways of anesthesia in PKP, and epidural anesthesia is also applied to PKP to some extent. However, all these three anesthetic methods have their respective advantages and disadvantages. It is essential to compare and evaluate the effects of different anesthesia methods on PKP for treating spinal fractures.

**Method:**

A total of 45 patients (53 vertebral bodies were included) were divided into two groups. Group A included 24 patients (29 vertebral bodies) with an average of 71 years old and Group B included 21 patients (24 vertebral bodies) with an average of 74 years old. Visual analogue scale (VAS) scores were recorded preoperatively; balloon expansion and bone cement injection were conducted intraoperatively. Then, they were recorded immediately after operation, 6 h postoperatively, to assess the pain level of the patient. Moreover, hospitalization time (days), operation duration (minutes), and bone cement injection amount (mL) had also been recorded.

**Results:**

There was no significant difference in preoperative general information and VAS score. However, the VAS scores were statistically significant at both the moment of balloon expansion and injection of bone cement. At the moment of immediate postoperation, the VAS scores showed no statistically significant difference, while it showed a statistically significant difference 6 h postoperatively.

**Conclusion:**

The anesthesia method by injection of 1% lidocaine hydrochloride (5 ml) into vertebral body can effectively relieve patients' pain in intraoperation and postoperation.

## 1. Introduction

With the aging of the population, industrialization of society, and the increasing rate of tumor diagnosis, the incidence of osteoporotic compression fractures, traumatic spine fractures, and pathological spine fractures in the elderly is increasing year by year. Among these types of fractures, compression fractures caused by senile osteoporosis are the most.

The article "Clinical Observation of Intraosseous Anesthesia in Percutaneous Kyphoplasty" was published in 2021. Journal: J Healthc Eng.

It is reported that there are about 200 million people with osteoporosis worldwide [1, 2], among which the most common is menopausal women over 50 years old [3], and the majority of osteoporotic fractures are vertebral fractures [4]. Furthermore, there are about 1.4 million people with vertebral fractures caused by osteoporosis worldwide [5, 6]. Among all fractures in all parts of the body, vertebral fracture accounts for about 5%–6%. Due to the special anatomical position, thoracolumbar spine fracture is the most common one, which accounts for over 90% [7].

Spinal fractures in the elderly as a high incidence of disease should not be ignored. Vertebral fractures often cause acute or chronic pain. In severe cases, they can cause kyphosis, which can limit daily activities and reduce quality of life [8, 9]. In the most serious case, it can be paralysis or even life-threatening, placing a heavy financial burden on the families of the patients [10–12].

Percutaneous kyphoplasty (PKP) is the minimally invasive surgery applied to the treatment of spinal fractures [13, 14]. PKP can effectively reduce low back pain, significantly reduce the length of hospital stay, restore Cobb angle, and improve sagittal plane sequence of patients [15, 16]. With the development of engineering technology, some scholars have found that adding a certain concentration of gold nanoparticles into nanocomposite cement can improve its punching resistance and antibacterial activity [17]. Scholars have shown that the three-dimensional scaffold composed of PCL matrix and iron oxide (Fe_3_O_4_) or iron-doped hydroxy-apatite (FeHA) nanoparticles can improve the modulus and yield stress of the fibers, as well as the modulus of the scaffold. Human mesenchymal stem cells (HMSCs) showed better adhesion and good spreading ability on PCL/Fe_3_O_4_ and PCL/FeHA nanocomposite scaffolds [18]. The emergence of new bone cement with the above characteristics is bound to further improve the curative effect of surgery.

The PKP is mainly performed with local anesthesia or general anesthesia [19]. Patients with general anesthesia have good tolerance during the operation and mechanical ventilation is convenient for breathing management under general anesthesia. Moreover, emergency rescue should be carried out quickly in critical situations such as bone cement embolism or allergy [20]. However, PKP under general anesthesia is associated with a high incidence of complications related to endotracheal intubation and respiratory depression [21]. Because the periosteum of the lateral pedicle and posterolateral vertebral body is rich in sensory nerves, it is very sensitive to painful stimulation. Under normal circumstances, the pain during local anesthesia is obvious, which is unbearable for some patients. Severe pain will increase the probability of intraoperative spinal cord and nerve injury and cause great psychological interference to patients. However, it has little effect on the trachea, and the patient has clear consciousness. If there are nerve complications caused by puncture, it can be detected in time [22]. It is a relatively common anesthesia method. Hannallah reported that intraspinal anesthesia was applied to PKP, and the puncture difficulties and injuries caused by hemodynamic fluctuations after anesthesia, spinal degenerative changes in the elderly, and spinal deformity caused by OVCF were problems that cannot be ignored in clinical practice [23].

The article "Clinical Observation of Intraosseous Anesthesia in Percutaneous Kyphoplasty" was published in 2021. Journal: J Healthc Eng.

Up to now, the choice of anesthesia method for PKP surgery is still a controversial topic. This paper will provide an important method for the anesthesia method for PKP surgery by comparing the analgesic effect of ordinary local infiltration anesthesia and intravertebral injection of anesthesia drugs.

## 2. Materials and Methods

### 2.1. Clinical Data

#### 2.1.1. The General Information

A total of 45 patients who were treated by PKP were selected from December 2016 to June 2017 in the spine surgery of the First Affiliated Hospital of Dalian Medical University, and all patients were divided into two groups. In group B, only the periosteum around the puncture point from the skin to the articular process joint was infiltrated with anesthetics layer by layer. The anesthesia method for Group A was injecting 5 mL of 1% lidocaine hydrochloride into the vertebra on the basis of anesthesia method of group B. Group A included 24 patients (10 male and 14 females) with 29 vertebral (thoracic 11, lumbar 18), which aged from 49 to 87 with an average of 71 years old. Group B included 21 patients (4 male and 17 females) with 24 vertebral (thoracic 6, lumbar 18), which aged from 49 to 96 with an average of 74 years old. All patients had preoperative pain of varying degrees without neurological injury, which was confirmed as a fresh fracture by MRI. PKP of bilateral pedicle puncture was performed on all patients, and X-ray, CT, MRI, and other related examinations were performed on all patients, which proved that there were no compression of the spinal cord in the spinal canal, nerve root compression, and no contraindications. There were a total of 29 patients with a history of falls before onset, 8 with bending sprain, and 8 with symptoms without obvious inducement. All patients completed the operation safely, obtained the informed consent of the patients before the operation, and obtained the approval of the ethics department of the hospital.

The article "Clinical Observation of Intraosseous Anesthesia in Percutaneous Kyphoplasty" was published in 2021. Journal: J Healthc Eng.

#### 2.1.2. Included Criteria

1. Patient with a medical history of a fall or of no definite history of trauma. And the patient was treated for chest, waist, and back pain.
2. During physical examination, there was no obvious nerve symptoms in the lower extremities except percussion pain in the injured vertebra.
3. X-ray and CT image criterion: vertebral body compression was wedge shaped; the posterior wall of the injured vertebra was not damaged; the spinal cord was not compressed, simple compression fracture or mild explosive fracture. Preoperative MRI showed low-signal changes in t1-weighted images, high signal in t2-weighted images, and lipid suppression images.
4. Etiology is the diagnosis of vertebral neoplastic diseases (such as metastatic tumors).

#### 2.1.3. Exclusion Criteria

1. Does not meet the above diagnosis
2. Patients with severe systemic diseases of the whole body, poor tolerance to surgery, and mental illness
3. Surgical site of skin inflammation, bleeding and other conditions, osteomyelitis, and allergic patients

#### 2.1.4. Therapeutic Effect Evaluation Index

During the operation, whether there was the leakage of PMMA, patients' vital signs' changes and emotional expressions were recorded. The following were recorded: the visual analogue scale (VAS) [24] before operation (on the surgery bed), intraoperative expanding balloon and injection of PMMA after operation (operation under the bed) and postoperative 6 hours to estimate the level of patient pain and compare the length of hospital stay (days), operation time (minutes), and PMMA injection quantity (ml) indicators of the two groups.

### 2.2. Surgical Method

#### 2.2.1. Surgical Materials

Operating system of PKP, concentration of 1% lidocaine hydrochloride injection (Suicheng Pharmaceutical Ltd.), ECG monitoring equipment, Siemens C arm and related protective equipment, sterile operating articles, etc.

#### 2.2.2. The Surgical Procedure

1. The pedicles on both sides were shown symmetrically on the C-arm X-ray machine. The position of the affected vertebral pedicle is marked on the body surface, and the lateral projection of about 4 mm of the outer edge of the vertebral pedicle is selected as the puncture point (Figure 1).
2. The operative region skin was disinfected and the area was draped. Lidocaine hydrochloride (1%) injection was used to local infiltration anesthesia lateral line about 4 mm outside the projection point. Then infiltration to the vertebral periosteum step by step and cutting a small incision in anesthesia needle were carried out (Figure 2).
3. Under C-arm fluoroscopy, a puncture needle was gradually inserted at the puncture position and a lateral radiograph showed the puncture needle reaching the trailing edge of the vertebral body. After puncturing 2-3 cm to the trailing edge of the vertebral body, the inner core of the puncture needle was taken out. Then, the guided needle was inserted into the puncture needle shell until 2-3 cm to the trailing edge of the vertebral body before taking out the puncture needle shell. The working channel along the guided needle 2-3 cm to the trailing edge of the vertebral body is shown in Figure 3.
4. All patients in group A were injected with 5 ml lidocaine hydrochloride injection (1%) at the external mouth of the right and left working channels. No drug was administered in group B (Figure 4).
5. The manual drill was used to enter the vertebral body along the working channel until the front end of the bit reached about 2-3 mm from the front edge of the vertebral body and pulled it out. The balloon was gently inserted into the vertebral body through the working channel. The balloon placed at 3/4 of the anterior vertebral body under the C-arm fluoroscopy's lower lateral position is well (Figure 5).
6. Contrast agent is gently injected into balloon under the perspective of C arm again and again, which makes the balloon expansion. Stopping injection until the vertebral's height restored satisfactorily or reaching the upper and lower end plate. The balloon was removed, and the dough stage bone cement was injected gently into the vertebral body under C-arm continuous perspective. Observing the bone cement's status, stopping injection until the bone cement leakage or the height of the vertebral body recovered satisfactorily (Figure 6).
7. The remaining bone cement inside the puncture needle sleeve was inserted into the vertebral body by inserting the needle core, and the sterile dressing was wrapped after local compression for 3-5 minutes at the puncture point for hemostasis. Three people raised stably the patient up to the flatcar, accompanied by doctors back to the ward.

The article "Clinical Observation of Intraosseous Anesthesia in Percutaneous Kyphoplasty" was published in 2021. Journal: J Healthc Eng.

#### 2.2.3. Observation Target

VAS scores of preoperation, expanding intraoperative balloon, injection of bone cement, end of operation and operation 6 hours later were collected. We also recorded intraoperative bone cement leakage, changes in patient vital signs and emotional expression, etc., and compared the indicators of hospitalization time (days), operation time (minutes), and bone cement injection (ml) of the two groups.

#### 2.2.4. Statistical Processing

In this study, SPSS18.0 was used for statistical analysis of the data. The measurement data were expressed by *x* ± *s*. The comparison between groups was performed by independent sample one-tailed *t*-test, and the count data was analyzed by *χ*^2^ test. The data of the two groups were compared in pairs, and the difference was statistically significant at *P* < 0.05.

## 3. Results

### 3.1. Comparison of General Condition between Two Groups of Patients

Both groups of patients completed the operation safely and smoothly. There were a few bone cement leaks in the two groups, and no neurological symptoms occurred. Some patients in group B screamed and even cried when they expanded the balloon during surgery. Some patients' heart rate and blood pressure suddenly increased during the expansion of the balloon and bone cement. The pain disappeared after stopping the operation. In group A, the vital signs during operation were relatively stable, and speech comfort was effective. There were no allergic reactions to lidocaine in all cases. All patients had a significant reduction in postoperative pain, could remove bed to exercise, and their X-ray cement's position was well on the first day after surgery. There were no statistically significant differences in gender and age between the two groups.

### 3.2. VAS Scores in the Two Groups Were Compared in Different Periods

There was no statistically significant difference in preoperative VAS scores between the two groups. The intraoperative balloon expansion VAS scores of group A and B were 7.28 ± 0.60 and 8.08 ± 0.50, respectively, with statistically significant difference (Table 1). The intraoperative injection of bone cement VAS scores of group A and B were 7.28 ± 0.76 and 8.17 ± 0.48, respectively, with statistically significant difference (Table 1). It indicated that intraoperative injection of lidocaine into the vertebral body can alleviate the pain caused by dilating the balloon and injecting bone cement to change the pressure in the vertebral body. The end of operation VAS scores of groups A and B were 2.46 ± 1.02 and 3.57 ± 3.94, respectively, with no statistically significant difference (Table 1). The possible reason was that the strength of the vertebra was increased and the fractured vertebra was stabilized reducing the stimulating effect on the internal nerves, after the vertebral body's height recovered. The 6 hours after operation VAS scores of groups A and B were 0.67 ± 0.64 and 0.67 ± 0.97, with statistically significant difference (Table 1). We supposed that the anesthesia method of intraoperative injection of lidocaine in the vertebral body could alleviate the patient's postoperative pain, but the mechanism was not clear.

### 3.3. The Hospitalization Time, Operation Time, and Injection Volume of Bone Cement Were Compared between the Two Groups

The hospitalization time (days) and operation time (minutes) of groups A and B were 5.96 ± 1.49, 6.10 ± 1.14 and 34.58 ± 8.96, 31.43 ± 7.93, respectively, but there was no statistical significance between the two groups (Table 1). The amount of bone cement injection (ml) in groups A and B was 9.35 ± 2.53 and 7.96 ± 1.55, respectively, but the difference was also not statistically significant (Table 1).

The article "Clinical Observation of Intraosseous Anesthesia in Percutaneous Kyphoplasty" was published in 2021. Journal: J Healthc Eng.

## 4. Discussion

Spinal fractures not only bring physical pain to the patient, but also lead to spinal deformities that can affect the mood of patients and even result in depression. And spinal deformity can also lead to decreased lung function, thoracic and abdominal volume reduction, limited capacity to exercise. PKP, as a newly emerging minimally invasive technique for the treatment of spinal fractures in recent years, has been increasingly favored by clinicians and patients due to its good analgesic effect, rapid recovery of movement, and other advantages [25–27]. The basic principle of PKP is to send special balloon percutaneous and pedicle into the fractured vertebral body and then restore the height of part of the vertebral body by expanding the balloon and injecting bone cement to stabilize the vertebral body, which finally can reduce the pain of patients. PKP is currently mainly performed under local infiltration anesthesia or general anesthesia, and epidural anesthesia has also been reported in literature. With the development of advanced analgesic theories [28] in recent years, increasing attention has been paid to the pain management of patients by medical staff.

### 4.1. Bone Cement Used in PKP Surgery

Self-polymerized polymethyl methacrylate (PMMA) is the most commonly used bone cement in PKP surgery. Infection is likely to occur with any intervention for spinal disease [29], and the main pathogen is methicillin-sensitive *Staphylococcus aureus*, but there is an alarming increase in the incidence of postoperative spinal infections that detect MRSA [30]. Infection after PKP is rare, but the consequences are serious [31]. In view of postoperative orthopedic infection, some scholars enhanced the antibacterial and antibiofilm activities of nanocomposite bone cement by adding gold nanoparticles (diameter 10e20 nm) to the modified bone cement samples through the in vitro effects of bacterial adhesion and proliferation [17]. In terms of vertebral height recovery, the stiffness of bone cement will directly affect the effect of PKP surgery. Some scholars skillfully used the magnetic characteristics of PCL/Fe_3_O_4_ and PCL/FeHA bone cement and quantified the addition of Fe_3_O_4_ and FeHA nanoparticles to increase the stiffness of bone cement [18]. In this study, traditional bone cement was used, and we will conduct further research on the new bone cement of the abovementioned scholars in a large sample.

The article "Clinical Observation of Intraosseous Anesthesia in Percutaneous Kyphoplasty" was published in 2021. Journal: J Healthc Eng.

### 4.2. PKP Analgesic Mechanism

Some scholars [32, 33] believe that the aggregation of bone cement generates heat dissipation to the tissues around the vertebra, which is enough to cause degeneration of proteins around the vertebra, cell necrosis, and nerve ablation. Other scholars [34, 35] believe that, in addition to the factors that lead to the necrosis of the peripheral nerve of the vertebral body caused by bone cement, the increased strength of the vertebral body reduces the stimulation of the fracture on the nerves in the vertebral body, thus playing a role in pain relief. Other analgesic mechanisms have also been suggested, such as bone cement blocking small local blood vessels in the vertebra, causing ischemia in surrounding tissues, and blocking the accumulation of inflammatory factors.

### 4.3. PKP Anesthesia Method Selection

The choice of anesthesia for PKP has always been a controversial issue. Foreign PKP mostly adopts general anesthesia [36], and some scholars [37] have pointed out that general anesthesia PKP surgery has the advantages of almost painless and more satisfactory postoperative vertebral height recovery, but the intraoperative neurological symptoms of patients cannot be accurately known, and there are relatively more complications of nerve injury. The hospitalization time of local infiltration anesthesia is short, and the postoperative complications are less than those of general anesthesia, but in the intraoperative pain of patients, it has always been a concern of the medical community. Intraoperative vital signs of some patients fluctuate greatly, resulting in increased surgical risk and unsatisfactory postoperative vertebral height reduction [38, 39]. Some scholars [40, 41] adopt the anesthesia method of local anesthesia combined with intravenous sedation and believe that percutaneous vertebroplasty under local anesthesia was safe and effective in pain control, and they also believe early postoperative leaving-bed movement reduced postoperative complications related to general anesthesia. Therefore, for some patients at high risk of general anesthesia, local anesthesia is a better choice. In this study, local anesthetic drugs were injected into the vertebra to effectively reduce the pain of patients during the operation, which may be a better anesthesia method. Although PKP under local anesthesia has some problems, it is still a better choice.

### 4.4. Local Infiltration Anesthesia of Nerves in Vertebra

The earliest concept of intraosseous anesthesia comes from Orlov, who proposed in 1960 that intraosseous anesthesia was used in the treatment of hand and finger surgery [42]. After that, Waisman et al. [43] further developed on this basis. They used intramedullary injection of lidocaine into the bone marrow cavity of the upper and lower limbs, which was satisfactory in anesthesia for orthopedic surgery, and then the concentration of lidocaine in the blood is determined to be much lower than its toxic value. This method of intramedullary anesthesia by local block anesthesia is simple in technique, effective in analgesic anesthesia and has less complications after operation. Studies by many scholars [44–47] have confirmed the existence of nerves in the vertebra, among which the sinus nerve plays a major role, and the local anesthetic plays an analgesic role by anesthesia of the sinus nerve. Sesay et al. [48] significantly reduced the pain of 84% of patients undergoing percutaneous vertebroplasty by injecting 1% lidocaine into the vertebral body and believed that lidocaine played an analgesic effect by blocking the pain sensation of local sinus nerve branch fibers in the vertebral body. By detecting the blood concentration of lidocaine in venous blood at different times, it was found that the highest blood concentration of lidocaine in the blood was still lower than its toxic dose. Lidocaine has been widely used in local anesthesia due to its excellent characteristics of rapid efficacy, long duration of action, wide safety range, and no irritation to tissues [49]. According to the literature, the maximum dosage of lidocaine is 7 mg/kg. Mild nausea and vomiting may occur when the blood concentration of lidocaine is > 5 ug/ml, but severe poisoning symptoms or even death may occur when the concentration of lidocaine is > 10 ug/ml. However, the intraoperative dose of lidocaine is far less than the toxic dose, and the concentration is not high, which ensures the safety of lidocaine in intraoperative use. Huang et al. [50] conducted PKP surgery on 84 patients (91 vertebral bodies) with osteoporotic compression fractures in 2015 by injecting local anesthesia into the vertebra and found that intravenous anesthesia can effectively relieve intraoperative pain and improve the surgical experience of patients. The results of this study are consistent with the above view that analgesic effects can be achieved by blocking nerves within the vertebral body.

The article "Clinical Observation of Intraosseous Anesthesia in Percutaneous Kyphoplasty" was published in 2021. Journal: J Healthc Eng.

With the deepening and development of PKP research, this research also deserves further improvement. Such as the composition of bone cement used in the experiment is mainly of methyl methacrylate (PMMA), some scholars' study [33] found that after the injection of PMMA in the vertebrae will produce larger heat, the vertebral body closed in the anterior department and the center temperature can reach 44∼113°C, the temperature inside the vertebral canal can reach 39∼57°C, and in the front, center of the vertebral body and spinal canal more than 50°C temperature lasted for 55 minutes, 8 minutes, and 25 minutes, respectively. Whether such a high temperature will change the drug properties of lidocaine and what will happen to the local metabolism of lidocaine require more and larger samples to verify.

## 5. Conclusions

The anesthesia method of vertebral body injection of lidocaine can effectively reduce the intraoperative and postoperative pain of patients, which not only has the advantages of local anesthesia, greatly reduce the operation time, postoperative complications related to general anesthesia are less, shorten the hospitalization time, and reduce the cost of hospitalization, but also to a certain extent reduces the intraoperative and postoperative pain of patients, so that the intraoperative vital signs of patients can be more stable and better communication and cooperation with the surgeon can exist.

## Figures and Tables

**Figure 1:** Operation position and puncture position.

**Figure 2:** Locating the puncture position on both sides.

**Figure 3:** Setting up the work channel.

**Figure 4:** Intravertebral injection of local anesthesia.

**Figure 5:** Inserting the balloon.

**Figure 6:** Injection bone cement.

**Table 1:** Comparison of indicators between the two groups.

Indicators	A (*n* = 24)	B (*n* = 21)	*t* (*x*^2^)	*P*
Sex (male/female)	10/14	4/17	2.674^△^	0.102
Age (years)	70.88 ± 9.93	74.00 ± 11.02	−1.001	0.906
The hospitalization time (days)	5.96 ± 1.49	6.10 ± 1.14	−0.343	0.229
Operation time (minutes)	34.58 ± 8.96	31.43 ± 7.93	1.243	0.207
Volume of bone cement injection (ml)	9.35 ± 2.53	7.96 ± 1.55	2.343	0.131
Preoperative VAS scores	7.46 ± 0.83	7.10 ± 0.83	1.460	0.505
VAS scores for intraoperative balloon expansion	7.28 ± 0.59	8.08 ± 0.50^※^	−5.286	0.048
VAS scores for intraoperative injection of bone cement	7.28 ± 0.75	8.17 ± 0.48^※^	−5.016	0.002
VAS scores for end of operation	2.46 ± 1.02	3.57 ± 3.94	−1.334	0.095
VAS scores for 6 hours after operation	0.67 ± 0.64	0.67 ± .97^※^	0.000	0.023

*Note*. All data were expressed as‾*x* ± *s*. △ represents *x*^2^ value; ^※^ represents *P* < 0.05.

## Data Availability

Data are available upon request to the corresponding author.
